The article "Effect of Perioperative Dexmedetomidine Anesthesia on Prognosis of Elderly Patients with Gastrointestinal Tumor Surgery" was published in 2022. Journal: Comput Math Methods Med.

# Effect of Perioperative Dexmedetomidine Anesthesia on Prognosis of Elderly Patients with Gastrointestinal Tumor Surgery

**DOI:** 10.1155/2022/7889372

**Published:** 2022-07-21

**Authors:** Lijia Guo, Yufei Liu, Meitan Wang

**Affiliations:** ^1^First Affiliated Hospital of Harbin Medical University, Harbin, 150000 Heilongjiang, China; ^2^Harbin Children's Hospital, Harbin, 150000 Heilongjiang, China

## Abstract

It was to investigate the influence of perioperative dexmedetomidine (DEX) anesthesia on the prognosis of elderly patients with gastrointestinal tumor (GIT) surgery. 90 patients who underwent laparoscopic radical gastrectomy for GIT were included. They were randomly divided into the experimental group (45 cases) with DEX+general anesthesia, and the control group (45 cases) with epidural anesthesia+general anesthesia. The indicators after surgery were compared between the two groups. The mean arterial pressure (MAP) was 74.8 ± 3.5 mmHg and the heart rate (HR) was 52.7 ± 8.2 beats/min^−1^ in the experimental group, significantly lower than those of the control group (*P* < 0.05). The Visual Analog Scale (VAS) scores of both groups decreased greatly associated to those before surgery (*P* < 0.05). The levels of cortisol (COR) and immune adhesion inhibitor (FEIR) in the experimental group were significantly dissimilar from those in the control group (*P* < 0.05). The tumor necrosis factor-alpha (TNF-*α*) was 96.4 ± 21.8 ng/L in the experimental group, observably lower than that in the control group (*P* < 0.05). The postoperative diamine oxidase (DAO) and D-lactate (D-lac) were 62.4 ± 9.3 *μ*mol/mL and 33.8 ± 7.2 ng/L, respectively, in the experimental group, much lower than those in the control group (*P* < 0.05). There were also significant differences in the initial recovery of bowel sounds, defecation, and total length of hospital stay (LOHS) between the groups (*P* < 0.05). DEX anesthesia had ideal sedative and analgesic effects, improving the prognosis of patients during surgery, and shortening the LOHS. Thus, it deserved a clinical application value.

## 1. Introduction

With the development of modern society, the population is gradually showing an aging trend, and the proportion of elderly patients undergoing surgeries is increasing. When people become old, various organs in the body undergo degenerative changes gradually, the defense ability is weakened, and the metabolic efficiency of the body is also reduced [1]. Treatment measures such as surgery and anesthesia are likely to cause a defensive stress response in the elderly. In addition, the cardiovascular system of elderly patients is weak. When a stress response occurs, the body activates the hypothalamus-pituitary-adrenal axis, resulting in a large secretion of stress hormones, and eventually leading to serious adverse reactions [2]. With increasing age, the body is gradually aging, and the probability of suffering from gastrointestinal tumor (GIT) increases. At present, the treatment of this disease is often surgery [3]. With the developing concept of fast recovery surgery, laparoscopic surgery has been promoted [4]. It has the advantages of high safety, less trauma to patients, easier postoperative recovery, and fewer complications. However, some researchers consider that carbon dioxide pneumoperitoneum is required during laparoscopic surgery, and carbon dioxide accumulates in the abdominal cavity for a long time, which may easily lead to an enlarged probability of postoperative pain of upper shoulder and abdomen in patients [5].

Some clinical studies have found that as the probability of pain after laparoscopic surgery increases, the probability of opioid use also increases. But the use of opioids will cause many adverse reactions, such as mental dependence, nausea and vomiting, constipation, and respiratory depression [6]. Some studies also suggest that opioids can affect the normal proliferation of lymphocytes, resulting in a decrease in cytokine secretion [7]. It was shown that opioids can reduce human immunity to a certain extent [8] as well, especially elderly patients are more prone to such adverse reactions. Therefore, laparoscopic surgery has a certain negative impact on the perioperative safety of the elderly. Because the elasticity of blood vessels in the elderly is poor, and the stress response will induce insulin resistance, some elderly people will have a rise of blood sugar. This will further aggravate the damage to blood vessels and lead to increased cardiovascular and cerebrovascular risks in elderly patients [9]. The blood exhibits a hypercoagulable state in stress response, which makes an increased probability of thrombosis [10]. For the body of elderly patients with GIT has always been in a state of chronic consumption, coupled with the continuous differentiation of tumor cells destroying normal cells, the immune function of the body is weakened [11]. Laparoscopic surgery is performed under the tissues, which is prone to infection after surgery, leading to increased postoperative mortality in elderly patients [12]. Other clinical studies have exposed that the probability of postoperative tumor recurrence in patients with GIT is closely related to their own immunocompetence [13].

Epidural anesthesia has a good postoperative analgesic effect. It can inhibit the conductions of sympathetic nervous excitation and noxious stimulation, so that the application of opioids can be reduced. This anesthesia method can also advance immune function and reduce the probability of stress response effectively [14]. However, for elderly patients, this anesthesia method is inconvenient to operate, has a large impact on hemodynamic status, is easy to widen the block plane, and has many postoperative complications tough to control [15]. Dexmedetomidine (DEX) is one of the *α*2 adrenergic receptor agonists with the effect of improving immune function, but its specific mechanism of action is not clear [16]. DEX can inhibit sympathetic nerve activity and adenylate cyclase and has good sedative and analgesic effects in clinical applications. It is conducive to maintaining hemodynamic stability without serious respiratory depression, so it is widely applied [17]. However, it also has some side effects. When the dose is enlarged, it may lead to adverse reactions such as xerostomia, bradycardia, and hypotension in patients [18]. Compared with epidural anesthesia, DEX anesthesia is easier to operate as it can be administered by intravenous infusion, with fewer postoperative complications that can be controlled easier.

Therefore, in this research, patients undergoing laparoscopic radical gastrectomy for GIT were selected. The patients were divided and given two different surgical anesthesia methods, respectively. Effect of DEX anesthesia on the prognosis of patients with GIT surgery was discussed, to further advance the therapeutic effect and provide reference for the clinical surgical treatment of GIT.

## 2. Research Methods

### 2.1. Research Objects

90 patients who underwent laparoscopic radical gastrectomy for GIT in the First Affiliated Hospital of Harbin Medical University from March 2020 to October 2021 were selected. These patients were randomly divided into the experimental group (45 cases) and the control group (45 cases). For patients in the former, DEX+general anesthesia was given, while epidural anesthesia+general anesthesia were given in the latter. There were 46 males and 34 females, aged 62-83 years old, with a mean age of 68.5 ± 3.8 years old. They weighted 52-71 kg, with a mean weight of 63.6 ± 6.4 kg. Inclusion criteria were as follows:

1. According to the standards of American Society of Anesthesiologists, the patients were in grade II or III
2. The patients had no history of other gastrointestinal surgery. Exclusion criteria were also enacted
3. Patients had severe cardiovascular, cerebrovascular, or respiratory diseases
4. Patients had severe liver and renal dysfunction
5. Patients suffered from endocrine and metabolic diseases
6. Patients had a history of mental illness
7. Patients got the second-degree atrioventricular block
8. Those were allergic to anesthetics
9. Those could not perform epidural puncture

### 2.2. Anesthesia Methods

Two hours before surgery, the patients in both groups were given with 375 mL of surgical energy drink orally. After being into the operating room, blood pressure, heart rate (HR), electrocardiogram, etc. were routinely monitored. During surgery, the goal-directed fluid therapy was performed according to the pulse pressure variation. The conventional general anesthesia induction was applied with sufentanil 0.4-0.5 *μ*g/kg, etomidate 0.2 mg/kg, and rocuronium bromide 0.6 mg/kg. Intravenous anesthesia was maintained, and propofol was pumped intravenously to the patient at 4-8 mg/kg/h, as well as remifentanil at 0.05-0.2 *μ*g/kg/min. On the foundation of general anesthesia, patients in the experimental group were pumped with 1.0 *μ*g/kg DEX for 10 min before anesthesia induction; it was also pumped as 0.5 *μ*g/kg half an hour before the end of the surgery. The control group was given epidural anesthesia, for which the patients took the left lateral position. The puncture space was selected according to the surgical site, with the depth of the catheter was 3.5 cm. Before the anesthesia induction, 5 mL of 2% lidocaine was given. 5 min later, the effect of anesthesia was blocked and the level of anesthesia were tested. 5 mL of 0.2% ropivacaine was given through epidural space injection at the start of surgery, followed by regular administration for 50 min/time.

### 2.3. Observation Indicators

The mean arterial pressure (MAP) and HR of the two groups of patients were recorded before and after surgery, respectively; venous blood was collected before and after surgery to detect stress indicators. Serum norepinephrine (NE) concentration and serum cortisol (COR) concentration were determined by enzyme-linked immunosorbent assay (ELISA). The rate of direct tumor erythrocyte rosette (DTER), an immune stress indicator, was detected; the determination method was expounded as follows. 0.1 mL of fresh serum from normal people and 0.1 mL of Ehrlich ascites cancer solution were mixed well and had a water bath at 37°C for 30 min. Normal saline was filled up, and the mixture was washed and then horizontally centrifugated (2000 rpm/min). After 5 min, 0.05 mL of erythrocyte suspension to be tested (washed 3 times, 1 × 10 mL) was added to mix well; then, water bath was performed again at 37°C for 30 min. After taken out, it was added with 0.1 mL of normal saline and mixed well; afterwards, 0.05 mL of 0.25% glutaraldehyde was also added for mixing. After horizontal smear and Wright's staining, tumor cells became blue, erythrocytes were in red, and a tumor cell with 3 or more erythrocytes was denoted as a rosette. With 100 tumor cells, the DTER rate was calculated. The immune adhesion inhibitor (FEIR) was determined by Guo's method. The time of the first anal exhaust, time of first defecation, and the recovery time of bowel sounds, the time to get out of bed, the Visual Analog Scale (VAS) pain score, respiratory depression, nausea and vomiting, and the total length of hospital stay (LOHS) after surgery were recorded.

### 2.4. Assessment of Cognitive Function

Criteria for postoperative cognitive dysfunction (POCD) were as below. According to the developer's suggestions, if the object had less than 12 years of education, 1 point was added to the total score, so as to adjust for the influence of culture. A score below 26 indicated POCD [19]. For the timing of the test, it was tested 7 days after surgery.

### 2.5. Detection of Inflammatory Factors

The tumor necrosis factor-alpha (TNF-*α*) and interleukin-6 (IL-6) were communal indicators of the degree of inflammation. D-lactate (D-lac) and diamine oxidase (DAO) were common indicators of intestinal permeability. Blood was drawn from the patients and centrifuged, then the supernatant was collected for testing. The contents of D-lac, DAO, TNF-*α*, and IL-6 in blood were determined strictly according to the instructions of the ELISA kit [20].

1. D-lac determination: 40 *μ*L of sample for direct determination

Firstly, before D-lac was determined, the D-lac kit needed to be put at room temperature for about 40 min. To use the reagent, it was shaken or oscillated gently, so as to keep the concentration uniform.

Secondly, the standard substance was diluted. Five centrifuge tubes were marked as S1, S2, S3, S4, and S5, respectively. The standard substance stock solution (480 *μ*mol/mL) was diluted into 5 different concentrations using the standard substance diluent, which were in 15 *μ*mol/mL, 30 *μ*mol/mL, 60 *μ*mol/mL, 120 *μ*mol/mL, and 240 *μ*mol/mL, respectively.

Thirdly, sample loading was made. The sample well to be tested, the blank well, and the standard well were set according to the relevant standards. The blank well could not be added with samples, biotin-labelled anti-D-lac antibody, and streptavidin-horseradish peroxidase (HRP); the remaining steps were the same. 40 *μ*L of samples was added to the sample wells to be tested; then, 10 *μ*L of anti-D-Lac antibodies and 50 *μ*L of streptavidin-HRP were added in turn. 50 *μ*L of different concentrations of standards was into the standard wells; because the biotin antibody had been integrated into the standards in advance, there was no need to add 50 *μ*L of streptavidin-HRP. When the samples were added, moving the wall of the wells should be avoided, and the samples were added to the bottom of the microplate reader. Gentle shaking was made to keep the reagent concentration uniform. After covered with sealing film, they were incubated at 37°C for 60 min.

Fourthly, the solution was confected in the following principles. The ratio of fresh medical double distilled water: concentrated washing solution was 30 : 1. It was shaken gently to keep the concentration uniform and then was put at room temperature for use.

Fifthly, washing. The sealing film was slowly peeled off, the liquid was discarded, and the remains was spin-dried. It was necessary to fill each well with the washing solution, and then placed for 30 seconds before discarding. It was repeated 5 times according to the above principles, and finally the ELISA plate was pat-dried with absorbent paper.

Sixthly, color development. 50 *μ*L of color developer A was added to each well in order; then, 50 *μ*L of color developer B was also added to each well. The plate was shaken gently to make the concentration of reagent uniform. The corresponding wells were placed at a temperature of 37°C and protected from light for the reaction for 10 min.

Seventhly, the reaction was terminated. As 50 *μ*L of terminating agent was added to each well, the reaction could be terminated (the color changed from blue at first to yellow.)

Eighthly, the optical density (OD) wanted to be measured at 450 nm of the microplate reader.

Ninthly, the sample content was calculated according to the prepared standard curve. The calculation equation was shown

(1) $$\begin{array}{c} y=a+bx+{cx}^{1.5}+{dx}^{2}+{ex}^{3}. \end{array}$$

Table 1 shows the D-lac concentrations of the standards, and Figure 1 shows the D-lac standard curve.

(2) DAO determination: 40 *μ*L was sampled for direct determination

Firstly, it was needed to put the DAO kit at room temperature for about 40 min before the determination of DAO. For using the reagent, it was shaken gently to make the reagent keep a uniform concentration.

Secondly, for dilution of standard substance, 5 centrifuge tubes were noticeable as S1, S2, S3, S4, and S5, respectively. The standard substance diluent was utilized to dilute the standard substance stock solution (480 *μ*mol/mL) into 5 different concentrations of 15, 30, 60, 120, and 240 *μ*mol/mL, respectively.

Thirdly, for sample loading, the following 3 wells were set depending on the relevant standards, which were the sample well to be tested, the blank well, and the standard well, respectively. Samples, biotin-labelled anti-DAO antibodies, and streptavidin-HRP could not be added into the blank well. 40 *μ*L of samples was added into the sample well to be tested, and 10 *μ*L of anti-DAO antibodies were added in sequence. The remaining steps were the same as above.

Table 2 shows the DAO concentrations of the standards, and Figure 2 shows the DAO standard curve.

(3) Determination of TNF-*α*: 40 *μ*L of serum was taken directly for testing

Firstly, it was needed to put the TNF-*α* kit at room temperature for about 40 min before the determination. For the use of the reagent, it should be shaken gently for a uniform concentration.

Secondly, the dilutions of standard substance were made. With 5 centrifuge tubes marked as S2, S3, S4, S5, and S6, the standard substance stock solution (640 *μ*mol/mL) was diluted with standard substance diluent into 5 different concentrations for use. These were in 30 *μ*mol/mL, 60 *μ*mol/mL, 120 *μ*mol/mL, 240 *μ*mol/mL, and 480 *μ*mol/mL, respectively.

Thirdly, for sample loading, the following 3 wells were set according to the relevant standards, namely, the sample well to be tested, the blank well, and the standard well. There was no sample, biotin-labelled anti-TNF-*α* antibody, and streptavidin-HRP was added into the blank well. 40 *μ*L of the sample was added to the sample well to be tested; then, 10 *μ*L of anti-TNF-*α* antibody was added in sequence. The rest of steps were the same as above.

Table 3 shows the TNF-*α* concentrations of the standards, and Figure 3 shows the TNF-*α* standard curve.

(4) IL-6 assay: serum homogenate was taken directly for testing

Firstly, before the assay of IL-6, the IL-6 kit needed to be placed at room temperature for about 40 min. The reagent should be surprised or oscillated gently for an even concentration.

Secondly, the standard substance was diluted. Five centrifuge tubes were denoted as S2, S3, S4, S5, and S6, respectively. With standard substance diluent, the standard substance stock solution (640 *μ*mol/mL) was diluted into 5 different concentrations of 20, 40, 80, 160, and 320 *μ*mol/mL, respectively.

Thirdly, 3 wells were set as the sample well to be tested, the blank well, and the standard well, respectively, for sample loading, according to relevant standards. The blank well could not be filled with samples, biotin-labelled anti-IL-6 antibody, or streptavidin-HRP. 40 *μ*L of the sample was added into the sample well to be tested, while 10 *μ*L of anti-IL-6 antibody was added in order. The rest of steps were the same as above.

Table 4 shows the IL-6 concentrations of standards, and Figure 4 shows the IL-6 standard curve.

### 2.6. Handling of Special Cases

The possible special circumstances during the experiment mainly comprised (severe) hypotension, (severe) bradycardia, and respiratory depression. HR and arterial blood pressure-based HR and blood pressure at rest 5 min after arterial puncture catheter placement were monitored. Bradycardia was defined as HR < 60 beats/min or less than the 20% of baseline value, and the treatment was a single intravenous injection of atropine 0.1-0.3 mg. Plain bradycardia was defined as HR < 50 beats/min or lower than 30% of the baseline value. For the treatment measures, intravenous injection of atropine 0.3-0.5 mg was given. Intermittent intravenous injection of isoproterenol 2-10 *μ*g was given when there was no obvious effect, and this case was excluded. Hypotension was defined as a decrease in systolic blood pressure > 20% of the baseline. Severe hypotension was defined as a decrease in systolic blood pressure > 30% of the baseline. If blood pressure fluctuated continuously for over 2 min, vasoactive drugs were utilized or the dose of aesthetic drugs was adjusted. Respiratory depression was defined as pulse oxygen saturation (SpO^2^) ≤ 90% under inhalation condition. In the event of respiratory depression, oxygen should be given through a mask timely, and artificial ventilation should be performed to assist respiration if necessary. If the above situation could not be better, the case was excluded from the experiment.

## 3. Statistical Methods

The statistical software SPSS 22.0 was used for processing in this research, and the measurement data were expressed as ($\bar{x}\pm s$). When the data were in normal distribution and the alteration was homogeneous, the *t*-test was adopted for comparisons between the two groups, and the repeated-measurement analysis of variance was used for the comparisons among multiple groups. The enumeration data were expressed as the number of cases (%), while the unordered classification data were expressed by the *χ*^2^ test. *P* < 0.05 was considered the condition of a statistically significant difference.

## 4. Research Results

### 4.1. The Detection Results of Hemodynamic Indicators

The hemodynamic test results of the two groups of patients suggested that, compared with preoperative levels, the MAP and HR of both groups were decreased, but the control group showed no significant change (*P* > 0.05). The MAP 74.8 ± 3.5 mmHg and HR 52.7 ± 8.2 beats/min^−1^ in the experimental group were remarkably lower compared with those before surgery and were also significantly lower than the 88.7 ± 10.2 mmHg and 60.2 ± 8.8 beats/min^−1^ in the control group. The differences above were all statistically significant (*P* < 0.05), which could be observed in Figure 5.

### 4.2. Comparison of Perioperative Stress and Immune Indicators between the Two Groups

As the stress and immune indicators were detected, it was shown that the levels of NE and DTER in the two groups did not change much compared with preoperative levels, and the differences were not statistically significant (*P* > 0.05). The COR was 104.9 ± 16.2 ng/mL in the experimental group and 104.6 ± 15.7 ng/mL in the control group, both of which observably increased compared to those before surgery with statistically significant differences (*P* < 0.05). The FEIR was 17.6 ± 2.1% in the experimental group and 17.2 ± 2.3% in the control group were greatly lower than those before surgery, showing the differences of statistical significance (*P* < 0.05). As presented in Figure 6, no significant difference was shown between the two groups (*P* > 0.05).

### 4.3. VAS Pain Scores

Before surgery, there was not a significant difference in VAS scores between two groups (*P* > 0.05). After surgery, the average VAS score of the experimental group was 4.7 ± 2 and that of the control group was 4.6 ± 2.3, significantly lower than those before surgery with differences of statistical significance (*P* < 0.05). No significant difference was between the groups (*P* > 0.05), which could be discovered in Figure 7.

### 4.4. Postoperative POCD Scores

Postoperative POCD evaluation was performed on the patients. The results illustrated that POCD occurred in both groups, with 6 cases in the control group and 4 cases in the experimental group. Although there were differences, which were not significant between groups (*P* > 0.05). More details were displayed in Figure 8.

### 4.5. Comparisons of IL-6 and TNF-*α* Levels in Serum before and after Surgery

There was no significant difference in IL-6 before and after surgery in the experimental group (*P* > 0.05). TNF-*α*96.4 ± 21.8 ng/L was highly lower than that before surgery, and the difference was of statistical significance (*P* < 0.05). Compared to the control group, postoperative TNF-*α*115.3 ± 24.6 ng/L, the difference was also statistically significant (*P* < 0.05) as presented in Figure 9.

Not a significant change was found in serum DAO and D-lac levels in the control group before and after surgery, without a difference of statistical significance (*P* > 0.05). The postoperative DAO was 62.4 ± 9.3 *μ*mol/mL, and D-lac was 33.8 ± 7.2 ng/L in the experimental group, observably lower than the preoperative levels with statistically significant differences (*P* < 0.05). In the control group, the postoperative DAO was 72.7 ± 15.2 *μ*mol/mL and D-lac was 38.2 ± 6.4 ng/L. The levels in the experimental group were considerably lower compared with those of the control, and the differences were proved to be statistically significant (*P* < 0.05) in Figure 10.

### 4.6. Other Indicators

The time of the first anal exhaust, the time of first getting out of bed for activities, the postoperative respiratory depression, and postoperative MAP were not significantly different between groups (*P* > 0.05). In the experimental group, the average postoperative recovery time of bowel sounds was 2.8 ± 0.7 d, the average time of first defecation postoperatively was 6.1 ± 1.8 d, the average LOHS was 17.9 ± 8.1 d, and 2 cases had vomiting reaction. In the control group, the average recovery time of bowel sounds, the average time of first defecation, and the average LOHS postoperatively was 3.9 ± 1.2 d, 7.4 ± 1.6 d, and 25.5 ± 8.6 d, respectively. There were 6 patients got vomiting in the control group. Each indicator was markedly higher compared to the experimental group, and the differences were thought of statistical significance (*P* < 0.05) (Figure 11).

## 5. Discussion

GIT has developed into a common digestive tract tumor nowadays, which has a serious impact on the life and health of human beings, especially the elderly. Epidural anesthesia can inhibit sympathetic nerve conduction and sympathetic nerve excitation, thereby reducing the synthesis of catecholamines. Epidural anesthesia can also inhibit the hypothalamic-pituitary-adrenal axis pathway, reducing the secretion of COR and improving immune function [21]. DEX, as an adrenergic receptor agonist, has the effect of inhibiting sympathetic nerve activity and maintaining hemodynamic stability. It exerts its analgesic effect intraoperatively and can reduce the inhibition of breathing. Patients are easier to be awakened, and it also has the effect of improving immunity, reducing the dose of anesthetic drugs, and antichilling as well as diuretic effects. It is often used in the perioperative period of patients with radical mastectomy for malignant GIT and can improve the quality of prognosis [22]. This work compared two anesthesia methods and analyzed the effect of DEX on the prognosis of elderly patients with GIT.

The results exposed that, compared with preoperative levels, MAP and HR in both groups decreased. The MAP of 74.8 ± 3.5 mmHg and HR of 52.7 ± 8.2 beats/min^−1^ in the experimental group decreased dramatically compared with those preoperatively. MAP of 88.7 ± 10.2 mmHg and HR of 60.2 ± 8.8 beats/min^−1^ in the control group were significantly lower compared to the experimental group with statistically significant differences (*P* < 0.05). It was suggested that DEX had a stabilizing effect on hemodynamic situation and could inhibit the increase in HR and MAP effectively in patients undergoing extubating surgery. Similar previous study has shown that DEX can reduce the occurrence of agitation during the recovery period in patients with tonsillectomy after general anesthesia and has obvious sedative and analgesic effects [23]. After surgery, the average VAS score of the experimental group was 4.7 ± 2 and that of the control group was 4.6 ± 2.3, which were significantly lower than those before surgery with differences of statistical significance (*P* < 0.05). There was not a significant difference between the two groups (*P* > 0.05). Two patients in the experimental group had vomiting reactions, while 6 patients in the control group had vomiting reactions. A study has also confirmed that DEX can reduce the stress response effectively, enhance immunity, and relieve postoperative pain and the incidence of adverse reactions in patients undergoing radical gastrectomy for gastric cancer [24]. This is consistent with the results of this work.

COR can be utilized to reflect the degree of stress in the body [25], and FEIR is an indicator that reflects the adhesion function of red blood cells [26]. Surgical treatment will lead to a certain degree of weakened immune function and inhibit the immune adhesion of red blood cells, so the body's ability to remove tumor cells will also be weakened. It is necessary to reduce the adverse effects of laparoscopic gastrointestinal surgery on the immune function of elderly patients by changing anesthesia methods and anesthetic drugs. It is also necessary to enhance the immunity of patients and reduce the probability of recurrence. This work showed that the COR was 104.9 ± 16.2 ng/mL and 104.6 ± 15.7 ng/mL of the experimental and control groups, respectively, significantly increased compared with those before surgery. The FEIR of the experimental group was 17.6 ± 2.1%, and the FEIR of the control group was 17.2 ± 2.3%, both of which were notably lower than that before surgery with great difference statistically (*P* < 0.05). Therefore, the application effect of DEX was better and it was worthy of promotion. At present, there is no unified standard for the optimal timing of POCD assessment. Generally, POCD can be divided into early, mid-term, and long-term cognitive changes. Within 1 week after surgery, it is the early POCD cognitive change, the mid-term cognitive change is within 3 months after surgery, and 1-2 years after surgery, it is the POCD long-term cognitive change. Some study has shown that the possibility of patient death within 3 months after surgery can be predicted by early POCD assessment [27], so it is of great significance to evaluate the POCD of patients within 1 week after surgery. In this work, it was assessed 7 days after the surgery. POCD occurred in both groups, with 6 cases in the control group and 4 cases in the experimental group. Although there was a difference, it was not significant between the groups (*P* > 0.05), perhaps because of the small sample size included. Thus, the effect of DEX could not be fully determined.

Studies have also proved that DEX can reduce systemic inflammatory response effectively in cases of elderly malignant GIT treated by laparoscopic surgery, which is conducive to the rapid recovery of patients after surgery [28]. This work demonstrated that the postoperative TNF-*α* of 96.4 ± 21.8 ng/L in the experimental group was memorably lower than that before surgery, showing the difference of statistical significance (*P* < 0.05). It was also statistically and greatly different from the postoperative TNF-*α* of 115.3 ± 24.6 ng/L in the control group (*P* < 0.05). It was suggested that DEX had an anti-inflammatory effect. A number of animal experiments have shown that DEX can significantly inhibit the excessive generation of inflammatory factors such as TNF-*α*, IL-1*β*, and IL-6 [29]. The postoperative DAO of 62.4 ± 9.3 *μ*mol/mL and D-lac of 33.8 ± 7.2 ng/L were much lower than those before surgery in the experimental group, which were statistically different (*P* < 0.05). Compared with the postoperative DAO of 72.7 ± 15.2 *μ*mol/mL and D-lac of 38.2 ± 6.4 ng/L in the control group, those in the experimental group were statistically lower (*P* < 0.05). Recent studies have suggested that stimulating vagal activity can play an important protective role in the intestinal barrier function damage triggered by inflammatory factors by regulating the cholinergic anti-inflammatory pathway [30]. In accumulation, not a significant difference was discovered in the time of the first anal exhaust, the first time to get out of bed, the occurrence of postoperative respiratory depression, and the postoperative MAP between two groups (*P* > 0.05). The average recovery time of postoperative bowel sounds, the average time postoperative first defecation, and the average total LOHS was 2.8 ± 0.7 d, 6.1 ± 1.8 d, and 17.9 ± 8.1 d, respectively, in the experimental group. Those were 3.9 ± 1.2 d, 7.4 ± 1.6 d, and 25.5 ± 8.6 d, respectively, in the control group. Each indicator was remarkably and statistically higher than that of the experimental (*P* < 0.05). Some study has also revealed that perioperative application of DEX can promote the recovery of gastrointestinal function and shorten the time of intestinal paralysis in patients with laparoscopic colorectal radical surgery [31]. It is consistent with the results of this work as well.

## 6. Conclusions

Through the comparison with epidural anesthesia, it was found that DEX anesthesia could improve postoperative stress response and immune function effectively and had ideal sedative and analgesic effects. It could also dismiss postoperative inflammatory response and reduce incidence of postoperative nausea and vomiting. Thus, the intestinal function of patients could be protected, and the LOHS of patients could also be shortened, which were beneficial to improve the prognosis of patients after surgery. It deserved a clinical application value. However, due to limited conditions, the included sample size was small, the study time was short, and some results showed no significant difference. The long-term prognosis of DEX anesthesia for patients with GIT surgery needed additional exploration. It illustrates that DEX can improve the intestinal permeability of patients and maintain the barrier function of the intestinal tract compared to epidural anesthesia.

## Figures and Tables

**Figure 1:** D-lac standard curve.

**Figure 2:** DAO standard curve.

**Figure 3:** TNF-*α* standard curve.

**Figure 4:** IL-6 standard curve.

**Figure 5:** Comparison of hemodynamic indicators. Compared with preoperative level, the difference was considered statistically significant, ^∗^*P* < 0.05. The same compared to the control group, ^#^*P* < 0.05.

**Figure 6:** Comparison of immune indicators. Differences of statistical significance compared to preoperative levels, ^∗^*P* < 0.05. ^#^*P* < 0.05 compared to the control group.

**Figure 7:** Comparison of VAS scores. The statistically significant difference in comparison with the preoperative levels and those in the control group, respectively, ^∗^*P* < 0.05, ^#^*P* < 0.05.

**Figure 8:** Comparison of occurrences of POCD.

**Figure 9:** Comparison of serum TNF-*α* and IL-6 levels. Compared to the preoperative levels and the control group, ^∗^ and # marked the difference of statistical significance as *P* < 0.05, respectively.

**Figure 10:** Comparison of serum DAO and D-lac levels. The differences were of statistical significance compared to preoperative levels and the control group, respectively, ^∗^*P* < 0.05, ^#^*P* < 0.05.

**Figure 11:** Comparisons of various indicators of postoperative gastrointestinal recovery.

**Table 1:** D-lac concentrations of the standards.

Concentrations (*μ*mol/mL)	Measured OD	Absolute OD
0	0.119	0
15	0.404	0.285
30	0.671	0.552
60	1.105	0.986
120	1.677	1.558
240	2.334	2.215

**Table 2:** DAO concentrations of the standards.

Concentrations (*μ*mol/mL)	Measured OD	Absolute OD
0	0.105	0
15	0.284	0.178
30	0.484	0.378
60	0.850	0.744
120	1.359	1.254
240	1.929	1.823

**Table 3:** TNF-*α* concentrations of the standards.

Concentrations (ng/L)	Measured OD	Absolute OD
0	0.056	0
30	0.337	0.281
60	0.571	0.515
120	0.971	0.915
240	1.594	1.538
480	2.586	2.530

**Table 4:** IL-6 concentrations of standards.

Concentrations (ng/L)	Measured OD	Absolute OD
0	0.060	0
30	0.376	0.316
60	0.656	0.596
120	1.109	1.049
240	1.822	1.762
480	2.933	2.873

## Data Availability

The data used to support the findings of this study are included within the article.
